# Method for Diagnosis of Acute Lymphoblastic Leukemia Based on ViT-CNN Ensemble Model

**DOI:** 10.1155/2021/7529893

**Published:** 2021-08-21

**Authors:** Zhencun Jiang, Zhengxin Dong, Lingyang Wang, Wenping Jiang

**Affiliations:** ^1^School of Electrical and Electronic Engineering, Shanghai Institute of Technology, 100 Haiquan Road, Shanghai, China; ^2^School of Electrical and Electronic Engineering, Shanghai Jiao Tong University, 800 Dongchuan Road, Shanghai, China

## Abstract

Acute lymphocytic leukemia (ALL) is a deadly cancer that not only affects adults but also accounts for about 25% of childhood cancers. Timely and accurate diagnosis of the cancer is an important premise for effective treatment to improve survival rate. Since the image of leukemic B-lymphoblast cells (cancer cells) under the microscope is very similar in morphology to that of normal B-lymphoid precursors (normal cells), it is difficult to distinguish between cancer cells and normal cells. Therefore, we propose the ViT-CNN ensemble model to classify cancer cells images and normal cells images to assist in the diagnosis of acute lymphoblastic leukemia. The ViT-CNN ensemble model is an ensemble model that combines the vision transformer model and convolutional neural network (CNN) model. The vision transformer model is an image classification model based entirely on the transformer structure, which has completely different feature extraction method from the CNN model. The ViT-CNN ensemble model can extract the features of cells images in two completely different ways to achieve better classification results. In addition, the data set used in this article is an unbalanced data set and has a certain amount of noise, and we propose a difference enhancement-random sampling (DERS) data enhancement method, create a new balanced data set, and use the symmetric cross-entropy loss function to reduce the impact of noise in the data set. The classification accuracy of the ViT-CNN ensemble model on the test set has reached 99.03%, and it is proved through experimental comparison that the effect is better than other models. The proposed method can accurately distinguish between cancer cells and normal cells and can be used as an effective method for computer-aided diagnosis of acute lymphoblastic leukemia.

## 1. Introduction

Leukemia is cancer with an extremely high fatality rate. It is a hematological malevolent tumor caused by the malicious cloning of immature white blood cells in the bone marrow. Leukemia can be further divided into acute leukemia and chronic leukemia. Chronic leukemia normally has a long onset period. While quite the opposite, without special treatment, the average survival period for acute leukemia is only three months. As a type of acute leukemia, acute lymphocytic leukemia is the most important kind of childhood leukemia, and it accounts for 25% of childhood cancers [1]. In more than 50 years of development, the treatment of acute lymphoblastic leukemia has made great progress. With special treatment at the early stage, the initial complete response rate can reach more than 70% [2]. Therefore, it is particularly important to diagnose acute lymphoblastic leukemia in the early stage of its onset. In general, the main diagnostic method for acute lymphoblastic leukemia is through morphology. When there are a large number of B-lymphoblast cells (cancer cells) in the bone marrow, it can be diagnosed as acute lymphoblastic leukemia [3]. Accurately distinguishing B-lymphoid precursors (normal cells) from cancer cells is the key to the diagnosis of acute lymphoblastic leukemia. However, under a microscope, cancer cells are very similar to normal cells that it is hard to classify them. 

Assisting in the diagnosis of diseases with computer vision technology is a promising research direction in recent years. In computer vision technology, image recognition through deep learning is one of the important methods. As one of neural networks used most frequently in deep learning, convolutional neural network (CNN) has strong self-learning ability, adaptive ability, and generalization ability. Traditional image recognition methods require manual feature extraction and classification, while CNN only needs the image data as an input of the network, and the self-learning ability of the network can complete the image classification [4, 5]. Nahid et al. used a multichannel convolution neural network to identify chest radiographs and diagnose pneumonia. The classification accuracy rate of chest radiographs reached 97.92%, which provided a very reliable detection method [6]. Daoud et al. combined the methods of deep learning for extracting image features and manual extraction for processing breast ultrasound images to classify breast tumors. The average accuracy rate of classification reached 96.1%, which meant breast cancer could be accurately detected by breast ultrasound images [7]. Yang et al. applied deep learning to the recognition of bladder cancer, and the recognition accuracy rate in practical application reached 83.36%, which was the same as that of medical experts, proving the effectiveness of deep learning in the diagnosis of bladder cancer [8].

Similarly, there are some researchers using computer vision technology to diagnose leukemia. Ahmed et al. used machine learning algorithms and convolutional neural networks to classify four types of leukemia, with the highest accuracy of 88.25% [9]. Boldú et al. proposed a machine learning method for diagnosing acute leukemia based on peripheral blood images. Colour clustering and mathematical morphology were used to segment the images, and then machine learning algorithms were used to classify six types of cells. The accuracy rate of cell classification reached 85.8%, and the correct diagnosis rate for leukemia reached 94% [10]. Kasani et al. combined two models of NASNetLarge and VGG19 to classify leukemic B-lymphoblast cells and normal B-lymphoid precursor cells with a classification accuracy rate of 96.58%, which can accurately diagnose acute lymphoblastic leukemia and proved that the ensemble model was more effective than a single network [11].

The transfer learning method has also been widely used in medical image classification in recent years. Alshazly et al. used transfer learning to train chest CT images to diagnose COVID-19 patients, obtained 92.9% accuracy rate on the COVID-19-CT dataset, and then used visualization technology to explain the model predictions clearly [12]. El-Khatib et al. used deep learning methods to diagnose skin lesions. They trained a variety of image classification models based on convolutional neural network through training methods of transfer learning to distinguish different types of skin lesions. The experimental result showed that this method had a better effect in diagnosing skin lesions [13]. Brodzicki et al. trained a convolutional neural network model to classify *Clostridioides difficile* bacteria cytotoxicity using transfer learning methods and achieved a classification accuracy rate of 93.5% on 369 images, with excellent recognition [14].

The models used in these studies are all based on convolutional neural networks (CNNs). Unlike these CNN models, which rely too much on convolutional layers, vision transformer is based on the transformer structure, which is a deep neural network based on the self-attention mechanism. Transformer structure was first applied in the field of natural language processing (NLP), and the researchers extended it to the field of computer vision. Compared with the CNN model, the model based on transformer structure performs better in image classification. Bazi et al. applied the vision transformer to remote sensing image classification and used the CutMix data enhancement method to test multiple remote sensing image data sets. The experimental results showed that the vision transformer classification accuracy rate of remote sensing images exceeds the CNN model [15].

In summary, it is of great significance to assist in the diagnosis of acute lymphocytic leukemia by classifying leukemic B-lymphoblast cells (cancer cells) and B-lymphoid precursors (normal cells). In this article, we propose the ViT-CNN ensemble model to assist in the diagnosis of acute lymphoblastic leukemia. The main contributions are as follows:

1. We propose the ViT-CNN ensemble model to distinguish cancer cells and normal cells. This is a model that uses two different methods to extract and combine features from cell images. This is the first time the vision transformer model and the CNN model have been combined to diagnose acute lymphocytic leukemia.
2. We propose a data enhancement method of difference enhancement-random sampling (DERS), which solves the problem of data set imbalance.
3. The ViT-CNN ensemble model has a classification accuracy rate of 99.03% for cancer cells and normal cells.
4. We compare the ViT-CNN ensemble model with the ordinary CNN model and other ensemble models and prove that the ViT-CNN ensemble model proposed in this article performs better in classification accuracy.

The second section presents the data set used in this article, the method of processing the data, the model used in this article, the loss function, and the optimizer. The third section presents the experimental process and experimental results of the proposed method, as well as the comparison results with other models. The full article is summarized in the fourth section.

## 2. Materials and Methods

### 2.1. Data Set

The data set used to build the diagnostic model is the ISBI 2019 data set [16–20], and 10661 cell pictures of 73 subjects were selected, including 7272 pictures of leukemic B-lymphoblast cells (cancer cells) from 47 all patients and 3389 pictures of B-lymphoid precursors (normal cells) from 26 healthy persons. These cells have been segmented from the microscopic images, and each cell picture is a real image after collection. Some staining noise and illumination errors generated during the collection process have been repaired to a large extent. As shown in Figure 1, the morphology of the two cells is very similar, so a professional oncologist will annotate the label of the image. The labels of normal cells images are positive samples, and the labels of cancer cells images are negative samples.

### 2.2. Difference Enhancement-Random Sampling

Directly training on an unbalanced data set can easily cause the model to fall into overfitting or cause the generalization ability of the model to be weak. In order to solve the problem of data imbalance, this article proposes a data enhancement method based on difference enhancement-random sampling (DERS). Suppose the unbalanced data set *D*, there are *a* images of category *A* and *b* images of category *B*, where *a* < *b*. *N* kinds of data enhancement are performed on category *A*, and *M* kinds of data enhancements are performed on category *B* so that the number of *a* × *N* and *b* × *M* are relatively close. Then *L* images are selected from *a* × *N* images of category *A*, and *L* images are selected from *b* × *M* images of category *B*, thus ensuring that the number of category *A* and the number of category *B* in the new data set are the same, so that the new data set becomes a balanced data set.

### 2.3. Data Processing

Figure 2 shows the number of normal cells and cancer cells in the data set. It can be seen that this data set is an unbalanced data set.

For the data set used in this article, there are two categories of cell images, which are images of normal cells and cancer cells. The number of images of cancer cells is more than twice the number of images of normal cells. We use the method of difference enhancement-random sampling to process the data set.

Three data enhancement methods of left and right flip, counterclockwise rotation 90°, and pixel matrix transpose are used to generate new cancer cells images. Six data enhancement methods of left and right, flipping up and down flip, counterclockwise rotating 90°, counterclockwise rotating 180°, counterclockwise rotating 270°, and pixel matrix transpose are used to generate new normal cells images. The examples of the generated images are shown in Figure 3.

The number of cancer cells images was 29,088, and the number of normal cells images was 23,702. A new data set is created with 20,000 images randomly drawn from two newly generated images. The new data set is a completely balanced data set.  Figure 4 shows the number of normal cells and cancer cells in the new data set.

Before training the model, the images need to be preprocessed. The original size of the cells images is 450 × 450, the size of the cells images is adjusted to 224 × 224, and the image is normalized to prevent overfitting of the model.

### 2.4. The Overall Flow of the Method

The method proposed in this article diagnoses acute lymphoblastic leukemia by distinguishing leukemic B-lymphoblast cells (cancer cells) images and B-lymphoid precursors (normal cells). After the data is preprocessed, two image classification models are trained by transfer learning. The symmetric cross-entropy loss function is selected as the loss function, the RAdam optimizer is selected as the optimizer. We combine the two models to ViT-CNN ensemble model based on the weighted sum method, it helps doctors realize computer-aided diagnosis. The process is shown in Figure 5.

### 2.5. Model

This section presents the ViT model and the CNN model used in the ViT-CNN ensemble model proposed in this article.

#### 2.5.1. Vision Transformer

Transformer structure is widely used in NLP (natural language processing) [21]. The vision transformer model is completely implemented based on the transformer structure without any CNN structure [22]. Transformer structure consists of a set of encoder components and a set of decoder components, whereas the vision transformer model is an image classification model and does not require a decoder. Therefore, there is only an encoder component in transformer structure of the vision transformer. The encoder component is composed of a stack of six identical encoders. Each encoder is composed of a multihead attention layer and a feed forward layer, and both layers contain the structure of residual connection and the structure of LayerNorm. The structure of an encoder component of the vision transformer is shown in Figure 6.

The multihead attention is a kind of self-attention structure, and it allows the model to pay attention to different aspects of information, as shown in formula (1)–formula (3) of multihead attention.

(1) $$\begin{array}{c} Q_{i}=QW_{i}^{Q},\\ V_{i}=VW_{i}^{V},i=1,\ldots ,8, \end{array}$$

(2) $$\begin{array}{c} {\text{head}}_{i}=\text{Attention}\left(Q_{i},K_{i},V_{i}\right),\;i=1,\ldots ,8, \end{array}$$

(3) $$\begin{array}{c} \text{MultiHead}\left(Q,K,V\right)=\text{Concact}\left({\text{head}}_{1},\ldots ,{\text{head}}_{8}\right)W^{o}. \end{array}$$

In these formulas, *Q* means the query vector, *K* means the key vector, *V* means the value vector, and *W* means the weight matrix.

The linear embedding layer is an important structure in the vision transformer model. The linear embedding layer divides the image into multiple patches and then flattens the patches into a one-dimensional tensor. After the patch embedding operation is completed, location embedding and class embedding are added and input into transformer encoder. After being output by the transformer encoder, it will go through an MLP head structure, which is composed of a fully connected layer and an activation function. The activation function used here is GELU (Gaussian error linear unit), and its formula is shown as follows:

(4) $$\begin{array}{c} \text{GELU}\left(x\right)=0.5x\left(1+\tanh\left(\sqrt{\frac{2}{\pi }}\left(x+0.044715x^{3}\right)\right)\right). \end{array}$$

After outputting through the MLP head structure, a classification task will be performed. The problem studied in this article is a two-class classification problem, so the final output category of the vision transformer model is changed to two categories. The model overview of the vision transformer model is shown in Figure 7.

#### 2.5.2. CNN Model

Convolutional neural network (CNN) is composed of convolutional layers, activation function, pooling layers, and fully connected layers. In the CNN classification models, the convolutional layer, the activation function, and the pooling layer constitute the feature extraction layer to extract the features, while the full connection layer forms a classification layer for classification [23, 24]. The pooling layer is a down-sampling operation to reduce the dimensionality of the extracted features while retaining important information of the features. The convolutional layer is the core structure of CNN, as shown in the following formula:

(5) $$\begin{array}{c} y\left(t\right)=\int_{-\infty }^{\infty }x\left(p\right)h\left(t-p\right)\text{d}p=x\left(t\right)*h\left(t\right). \end{array}$$

In this article, EfficientNet is selected as the CNN model. EfficientNet is an image classification model proposed by the Google team in 2019 [25]. It is known as the strongest image classification model today. The EfficientNet model balances resolution, depth, and width to optimize efficiency and accuracy. The main idea of the EfficientNet is that all convolutional layers of a convolutional neural network must be uniformly expanded by the same proportional constant. The EfficientNet model uses MBCConv in MobileNet V2 as the backbone network of the model and uses the squeeze and excitation method in SENet to optimize the network structure. EfficientNet has eight versions of models, and this article uses the EfficientNet-b0 model. The original model has 1000 classifications, and this article has improved the original model, redesigned the classification layer, and improved its final output category to two categories. The structure of the EfficientNet-b0 model is shown in Figure 8.

### 2.6. ViT-CNN Ensemble Model

The ensemble model is a method to improve the accuracy rate of the model [26, 27]. The greater the differences between the models, the greater the performance improvement after the ensemble. Two different feature extraction methods extract the features of cell images, which can more comprehensively distinguish the differences between images and obtain better classification results. The ViT-CNN ensemble model combines two completely different feature extraction methods, vision transformer model and CNN (EfficientNet) model, to extract the features of cells images and classify them. The ensemble model method used in this article is the weighted sum method. The output results of the vision transformer model are multiplied by a coefficient of 0.7, and the output results of the EfficientNet model are multiplied by a coefficient of 0.3, and then the two results are added up together as the final prediction result.

### 2.7. Transfer Learning

Transfer learning solves the shortcoming that deep learning needs numerous samples to train models. The pretraining model obtained by training on large data sets can be trained with a few data sets, and the training time required for deep learning is greatly shortened. Fine-tuning is a kind of transfer learning method, and it takes the weight of the pretraining model as the initial weight and trains on the basis of the initial weight without training the model from scratch. Fine-tuning not only increases the convergence speed and generalization ability of the model but also reduces the risk of overfitting [28–30]. In this article, both the ViT model and the CNN model are trained by the method of fine-tuning of transfer learning.

### 2.8. Symmetric Cross-Entropy Loss Function

For medical images data sets, a bit of noise is unavoidable. The morphological similarity of cancer cells and normal cells results in some noise on the label. The symmetric cross-entropy loss function can reduce the influence of noise and prevent overfitting [31]. The definition of the symmetric cross-entropy loss function is shown as follows:

(6) $$\begin{array}{c} l_{\text{sce}}=l_{\text{ce}}+l_{\text{rce}}. \end{array}$$

Among them, *l*_ce_ is the cross-entropy loss function and *l*_rce_ is the reverse cross-entropy function. Its definition is shown as follows:

(7) $$\begin{array}{c} l_{\text{rce}}=-\sum_{k=1}^{K}p\left(k|x\right)\log\;q\left(k|x\right). \end{array}$$

Therefore, the symmetric cross-entropy loss function is used in this article as the loss function of the model to reduce the influence of noise on the generalization ability of the model.

### 2.9. Optimizer

RAdam optimizer is a new optimizer based on the classic Adam optimizer. In the training process of the model, the initial learning rate is very important. The Adam optimizer has too large variance and more uncertain factors, which leads to its insufficient stability. The RAdam optimizer is based on the Adam optimizer, which aims to introduce a correction to the adaptive learning rate to correct the variance of the Adam optimizer [32]. Compared with SGD optimizer and Adam optimizer, SGD optimizer has better convergence effect but slow convergence speed and Adam optimizer has fast convergence speed but easily converges to the local optimal solution. RAdam optimizer has good performance in convergence effect and convergence speed and is relatively compared with Adam optimizer, and it can stably improve accuracy.

## 3. Results and Discussion

### 3.1. Experiment Platform

The experimental platform used in this article includes a hardware environment, which consisted of Intel Core i7-9700f processor, NVIDIA RTX2060s 8 GB graphics card, and 16 GB memory. The proposed model is implemented in python3.7 using PyTorch [33] framework.

### 3.2. Performance Metrics

There are many evaluation indicators for image classification, but for the problem of assisting diagnosis of cancer through image classification, accuracy and precision of the classification model play a significant role. Therefore, accuracy and precision are selected as the indicator for evaluating the performance of the proposed model. The accuracy rate is defined as the ratio of correctly recognized positive samples and negative samples to total samples, as shown in the following formula:

(8) $$\begin{array}{c} \text{ACC}=\frac{\left(\text{TP}+\text{TN}\right)}{\text{TP}+\text{TN}+\text{FP}+\text{FN}}. \end{array}$$

The precision rate is the ratio of correctly recognized positive samples to all positive samples, as shown in the following formula:

(9) $$\begin{array}{c} \text{precision}=\frac{\text{TP}}{\text{TP}+\text{FP}}. \end{array}$$

In the above formulas, TP is the samples predicted to be positive samples in the positive samples, TN is the samples predicted to be negative samples in the negative samples, FP is the samples predicted to be positive samples in the negative samples, and FN is the samples predicted to be negative samples in the positive samples.

### 3.3. Experimental Comparison

The implementation process of the method proposed in this article is as follows:

 
*Step 1*. The new balanced data set is divided into training set, validation set, and test set at a ratio of 8 : 1 : 1
 
*Step 2*. The learning rate is set to 0.0001, the training batch size is set to 32, and the validation batch size is set to 32
 
*Step 3*. The vision transformer model is trained for 30 epochs, and then the parameter model with the highest accuracy is saved in the validation set
 
*Step 4.* The EfficientNet model is trained for 30 epochs, and then the parameter model with the highest accuracy is saved in the validation set
 
*Step 5*. The vision transformer model and the EfficientNet model are integrated into the ViT-CNN ensemble model for testing

The experiment is carried out according to the above procedure. The loss change curve of the training set and the accuracy change curve of the validation set of the vision transformer model and the EfficientNet model are shown in Figure 9.

The accuracy rate and the precision rate of the vision transformer model, the EfficientNet model, and the ViT-CNN ensemble model on the test set are shown in Table 1.

As can be seen from Table 1, the accuracy rate of the vision transformer model is 3.72% higher than that of the EfficientNet model and the precision rate of the vision transformer model is 1.52% higher than that of the EfficientNet model, and those showed that the performance of the vision transformer model is better than the performance of the EfficientNet model. After being ensemble into the ViT-CNN ensemble model, the accuracy rate reached 99.03%, the precision rate reached 99.14%, and the performance is further improved.

The accuracy rate can judge the classification ability of the model, but the specific details cannot be reflected. The confusion matrix is the comparison matrix between the predicted result and the actual value, which can clearly indicate the prediction details of each category when the classification model is making predictions. The confusion matrix is used to further analyze the classification ability of the ensemble model proposed in this article. The confusion matrix of three models is shown in Figure 10.

It can be seen from the confusion matrix that the recognition ability of the vision transformer model is very balanced, with the recognition accuracy of cancer cells and normal cells as the same. The EfficientNet model has a difference in the ability to recognize cancer cells and normal cells, and the ability to recognize cancer cells is stronger. The ViT-CNN ensemble model has the same recognition accuracy for normal cells as the vision transformer model but has a stronger ability to recognize cancer cells. In practical applications, better identification of cancer cells can more accurately diagnose acute lymphocytic leukemia, so the ViT-CNN ensemble model can in a superior way assist in the diagnosis of acute lymphocytic leukemia.

In order to prove the effectiveness of the method, the proposed model in this article is compared with the following models:

1. *Other CNN Models*. This article compared the ViT-CNN ensemble model with Resnet50, Densenet121, and VGG16 three classic CNN models.
2. *Model in Literature* [11]. Literature [11] has the best current research results on diagnosis of acute lymphoblastic leukemia. This article compared the accuracy of the model they proposed.

The specific comparison is shown in Table 2.

It can be seen from Table 2 that the accuracy rate of the ViT-CNN ensemble model is 4.08%, 5.38%, and 3.79% higher than the accuracy rate of the Resnet50, Densenet121, and VGG16. This shows that the ViT-CNN ensemble model has a better ability to classify cancer cells and normal cells. Compared with the model in literature [11], the accuracy rate of the model proposed in literature [11] is 96.58%, while the accuracy rate of the ViT-CNN ensemble model is 99.03%; this accuracy rate is 2.45% higher than the model proposed in the literature. Obviously, the ViT-CNN ensemble model has better classification performance and can assist in the diagnosis of acute lymphocytic leukemia more accurately.

## 4. Conclusions

In this article, we proposed a diagnostic approach for acute lymphocytic leukemia, which could classify cancer cells and normal cells through an ensemble model to assist doctors in the diagnosis in reality. The ISBI 2019 data set was used in the article; we proposed the difference enhancement-random sampling (DERS) method to solve the problem of data imbalance. We designed an ensemble model that integrates the vision transformer model and the EfficientNet model into the ViT-CNN ensemble model. The accuracy of this model in the classification of B-lymphoblastic cells and normal B-lymphoid precursors was 99.03%. We compared the ViT-CNN ensemble model with Resnet50, Densenet121, and VGG16 three classic convolutional neural Nnetwork models. The ViT-CNN ensemble model significantly outperformed these previous models. The results showed that the model proposed in this article was superior to other models in accuracy and had a balanced classification ability, which could better assist in the diagnosis of acute lymphoblastic leukemia.

## Figures and Tables

**Figure 1:** (a) Normal cells. (b) Cancer cells.

**Figure 2:** The number of normal cells and cancer cells.

**Figure 3:** The examples of the generated images: (a) cancer cells; (b) normal cells.

**Figure 4:** The number of normal cells and cancer cells in the new data set.

**Figure 5:** The process of the method.

**Figure 6:** The structure of an encoder component of the vision transformer.

**Figure 7:** The model overview of the vision transformer model.

**Figure 8:** The structure of the EfficientNet-b0 model.

**Figure 9:** Loss change curve of training set and accuracy change curve of validation set. (a) Train loss of the vision transformer model. (b) Val accuracy of the vision transformer model. (c) Train loss of the EfficientNet model. (d) Val accuracy of the EfficientNet model.

**Figure 10:** Confusion matrix of three models: (a) the vision transformer model; (b) the EfficientNet model; (c) the ViT-CNN ensemble model.

**Table 1:** The accuracy and precision of three different models.

Model	Accuracy (%)	Precision (%)
Vision transformer	98.90	98.90
EfficientNet	95.18	97.38
ViT-CNN ensemble model	99.03	99.14

**Table 2:** The comparison of accuracy of five different models.

Model	Accuracy (%)
Resnet50	94.95
Densenet121	93.65
VGG16	95.24
Model in literature [11]	96.58
ViT-CNN ensemble model	**99.03**

## Data Availability

The data used in this work are from public datasets: ISBI 2019 C-NMC Challenge: Classification in Cancer Cell Imaging (https://competitions.codalab.org/competitions/20395). To apply for the access to dataset, a registration is required.
